# Advancing the Regulation of Traditional and Complementary Medicine Products: A Comparison of Five Regulatory Systems on Traditional Medicines with a Long History of Use

**DOI:** 10.1155/2021/5833945

**Published:** 2021-10-27

**Authors:** Zuanji Liang, Hao Hu, Junlei Li, Dongning Yao, Yitao Wang, Carolina Oi Lam Ung

**Affiliations:** Institute of Chinese Medical Sciences, State Key Laboratory of Quality Research in Chinese Medicine, University of Macau, Macao, China

## Abstract

**Background:**

An appropriate regulatory system to ensure and promote the quality, safety, and efficacy of the products of traditional medicine (TM) and complementary medicine (CM) is critical to not only public health but also economic growth. The regulatory approach and evaluation standards for TM/CM products featured with a long history of use are yet to be developed. This study aims to investigate and compare the existing regulatory approaches for TM/CM products with a long history of use.

**Method:**

A mixed approach of documentary analysis involving official and legal documents from official websites, as well as a scoping review of scholarly work in scientific databases about regulatory systems of TM/CM products in China, Hong Kong, Taiwan, Japan, and Korea, was employed in this study and used for comparison.

**Results:**

For registration purposes, all five regulatory systems recognized the history of use as part of the totality of evidence when evaluating the safety and efficacy of TM/CM products with a long history of use. Generally, the list of classic formulas is predefined and bound to the formulas recommended in the prescribed list of ancient medical textbooks. Expedited pathways are usually in place and scientific data of nonclinical and clinical studies may be exempted. At the same time, additional restrictions with the scope of products constitute a comprehensive approach in the regulation. Quality assurance and postmarketing safety surveillance were found to be the major focus across the regulatory schemes investigated in this study.

**Conclusion:**

The regulatory systems investigated in this study allow less stringent registration requirements for TM/CM products featured with a long history of use, assuming safety and efficacy to be plausible based on historic use. Considering the safety and efficacy of these products, regulatory standards should emphasize the technical requirements for quality control and postmarket surveillance.

## 1. Introduction

Traditional medicine (TM) and complementary medicine (CM) refer to a group of healthcare practices approaches that may be integrated into the mainstream healthcare system to various extent depending on the theories, beliefs, experiences, and culture indigenous to the population [1]. TM/CM are important if they are not the only health resources for treatment of major diseases, prevention and management of chronic conditions, and meeting the health needs of aging populations [2, 3]. While TM/CM refer to modalities that encompass both products or practices, the primary focus of this study is on the TM/CM products and the recent development in the regulatory landscape.

Across the globe, over 80% of the world's population use some form of TM/CM products and the trend is on the rise [4]. A preference for “natural or holistic” approach, a desire for a high degree of autonomy in self-management, and a perception of absolute safety contribute to the increasing use of TM/CM products [5, 6]. Indeed, growing evidence continues to show the benefits of TM/CM products in disease management in such cases as cancer, noncommunicable diseases [7, 8], and other serious illnesses [9–12]. The potentials of TM/CM products in managing pandemics such as severe acute respiratory syndrome [13] and coronavirus disease (COVID-19) [14–16], achieving universal health coverage [17, 18], and improving the overall quality of healthcare services [19] further underpin the importance of ensuring public health through effective regulatory measures [20, 21].

TM/CM products also have important economic implications. The global market for such products is expected to reach US $5 trillion by 2050 growing at an annual rate of 7% [22]. Significant expenditure has been reported in Asia-Pacific and such countries as United States, United Kingdom, and Canada [23–27]. In Australia, CM products represent a US $3.97 billion fast-growing industry, featuring 148 manufacturing sites, 2,852 direct employees, and US $311 million economic value [28]. In China, the total output value of the TM industry was US $122.4 billion or nearly one-third of the total output by the overall pharmaceutical industry, representing a new force driving the national economy growth [29]. Considering the above, an appropriate regulatory system to ensure and promote the quality, safety, and efficacy of such products is therefore critical to not only the quality of life but also economy growth.

The level and form of regulatory measures of TM/CM products lie on the recognition of the totality of evidence and the relevance of historical use in justifying the safety and efficacy. Arguably, both scientific knowledge and traditional knowledge are critical to informing the risk-based approach that ensures a balance of regulatory burden and product accessibility. For instance, the Therapeutic Goods Administration in Australia acknowledges the value of historical use when approving CM products listed in pharmacopeia or traditional medical literature [30]. The European Medicines Agency allows a simplified licensing system for TM products which have been proven to have historical use of 30 years or more in the European Union [31]. In China, the need for clinical safety data may be exempted for “classic Chinese medicine formulas” which have been used in clinical practice for hundreds or thousands of years [29, 32]. However, such risk-based regulatory approach is not necessarily the case in places where a full evaluation mechanism for TM/CM products is yet to be established.

According to the World Health Organization (WHO), as of 2018, only 124 Member States (64%) reported that they had laws or regulations on TM/CM products and there is not yet a standard approach in assessing the totality of evidence when evaluating the safety and efficacy of such products [3]. Recently, the concept *classic formula* featured with a long history of use has been introduced as a new regulatory category of the regulatory framework of TM/CM in countries or regions like China and Macao. However, little research has been conducted to systemically analyze the regulation standards of TM/CM products with a long history of use across the countries. Considering the regulatory need and the general quest for developing a reasonable regulatory system for TM/CM products with a long history of use, this study aims to investigate the existing regulatory approaches that adopt the concept of risk-based approach to TM/CM products with a long history of use and to illustrate a comparison. The study findings will help improve the understanding about the global regulatory landscape for TM/CM products and inform the formulation of technical requirements for the registration approval of TM/CM products.

## 2. Materials and Methods

### 2.1. Study Approach

For the purpose of this study, there is a need for a workable method to analyze and study the pharmacogovernance with a scientific and academic approach. A stepwise approach of (1) problems or need identification, (2) options formulation, (3) selected options adoption, (4) options implementation, and (5) outcome evaluation of implemented options was considered appropriate [33] and was thus proceeded accordingly. First, the need was determined to be the formulation of a set of regulatory requirements applicable to TM/CM products with a long history of use. Subsequently, the literature on regulating TM/CM products with a long history of use was consulted. While each drug regulatory authority has autonomy in adopting regulatory mandates deemed most compatible with the local requirements, it is also relevant to consider benchmarking regulatory models and sharing best practices [34]. For this, regulatory system comparisons were necessary to better inform and facilitate improvements if conducted among systems that share common challenges in their respective regulatory landscapes.

### 2.2. Study Targets

In this study, countries/regions were selected for comparison because they had already established registration processes for TM/CM products with a long history of use. In East Asian countries, traditional Chinese medicine (TCM) is known to have originated in China about 3,000 years ago [35]. It was introduced to Japan along with the entirety of the Chinese culture [36] and to Korea with Buddhism in the beginning of the 6^th^ century [37]. Before Western culture was introduced to East Asia in 19^th^ century, TCM was the main medical system used to treat all types of diseases [38] with some TCM decoction formulas still in use such as Shegan Mahuang Decoction recorded in “Synopsis of Golden Chamber” for asthma [39], Bu Zhong Yi Qi Decoction (Hochuekkito) recorded in “Spleen Gastric Theory” for infirmity [40–42], and Mahuang Decoction (Maoto) recorded in “Treatise on Fevers” for flu [43, 44]. Considering that China, Hong Kong, Taiwan, Korea, and Japan share the same TCM origin and regulatory interests in TM/CM products with a long history of use, they were included in this comparative study.

### 2.3. Data Collection and Analysis

A mixed approach of documentary analysis involved official and legal documents from official websites, as well as a scoping review of scholarly work in scientific databases about regulatory systems of TM/CM products. The official websites of the drug regulatory authorities in the selected countries/regions were searched for official documents (Table 1). Additionally, databases (Google Scholar, PubMed, Web of Science, and Chinese National Knowledge Infrastructure) were also searched and reviewed for TM/CM products regulation to supplement and improve the understanding of the regulation information collected from the above-mentioned official websites. The sensitive search terms used included the following: (herbal medicine^*∗*^ OR traditional medicine^*∗*^ OR traditional Chinese medicine^*∗*^) AND (regulation OR registration) AND (China OR Japan OR Korea OR Hong Kong OR Taiwan). Documentary analysis was employed to gather information about the TM/CM product regulatory approaches in selected countries/regions [45]. Information about the overall regulatory approach, listing of product formulas, major requirements and constraints for registrations, quality control requirements, and postmarket surveillance was extracted and used for comparison.

## 3. Results

### 3.1. The Overall Regulatory Approaches for TM/CM Products with a Long History of Use

Considering the differences in risk-based approaches adopted by the drug regulatory authorities, there is a great variation in terms of the definitions, the scope, and the corresponding regulatory approaches associated with TM/CM products featured with a long history of use in selected countries and regions. An overview of these regulatory frameworks for classic Chinese medicine formulation (CCMF) in China, established medicine in Hong Kong, standard formulation of Chinese medicine (SFCM) in Taiwan, Kampo medicine in Japan, and herbal drug in Korea is described in the following and summarized in Table 2.

#### 3.1.1. China

In China, TM/CM products are mainly divided into four registration categories, namely, innovative Chinese medicines, modified new Chinese medicines, generic Chinese medicines (same name and formulations), and CCMF [46]. Of particular interest in this study were CCMF, which featured a long history of use and were thus subject to evaluation that considered the totality of evidence. In 2017, the NMPA (known as the China Food and Drug Administration at the time) announced the draft of the Regulations of the Simplified Registration and Approval Management for CCMF [52]. The CCMF in this document referred to those listed on the ancient classic Chinese medical books prior to 1911 and conformed with the same stringent examination, regulation model, and approval standards as other medications in China since the implementation of “Provisions for Drug Registration” [53] in 1985. Accordingly, the adoption of a simplified registration and approval arrangement for CCMF was proposed. Considering the fact that CCMF already had their clinical effects demonstrated by hundreds of years' clinical application, clinical studies to demonstrate acceptable efficacy and safety would not be applicable as it would be for modern biochemical drugs.

#### 3.1.2. Taiwan

The TCM products management in Taiwan adopts two registration categories differentiated by the characteristics and the experiences of historical use. For TCM products that are traditional formulas listed in the classic TCM literature or known as the SFCM, registration and licensing may be approved in the absence of clinical efficacy/safety data according to the “Regulations for Registration of Medicinal Products” [47, 54]. SFCM is selected by the Chinese Medicine Association from the well-established publications and ancient classic medical books, of which the dosage form and formula contents have been standardized uniformly. These well-established publications [47] include a range of Chinese medicine bibliographies such as “Yi Zong Jin Jian (Golden Mirror of Medicine),” “Yi Fang Ji Jie (Analytic Collection of Medical Formulas),” and “Ben Cao Gang Mu (Compendium of Materia Medica).” However, when TCM products listed in the well-established publications are to be applied for new indications or new administrating routes, data about clinical efficacy is required for further evaluation. For TCM products not listed in the well-established publications, comprehensive documents in respect of safety, efficacy, and quality are required for registration application.

#### 3.1.3. Hong Kong

According to the Chinese Medicine Ordinance, under the broad term of “proprietary Chinese medicine” (any proprietary product composed solely of Chinese herbal medicines formulated in a finished dose form known or claimed to be used for disease or symptom management or functional state regulation of human body), there are 3 categories: the “established medicine,” the “nonestablished medicine,” and the “new medicine” [48]. Featured with a long history of use, “established medicine” refers to an ancient prescription originating from Chinese medicine bibliographies or well documented in Pharmacopoeia of the People's Republic of China (PRC) or the National Drug Standards of PRC [48]. There is a tiered regulation approach to “established medicine,” namely, Group I, Group II, and Group III. For Group I “established medicine,” only basic documents are required to demonstrate safety, efficacy, and quality when applying for registration. Additional evidence for safety and quality such as real-time stability test is required for Group II “established medicine,” while comprehensive documents including principal pharmacodynamic and clinical trial studies are applicable to Group III “established medicine” application.

#### 3.1.4. Japan

TM/CM products in Japan are crude drug products derived from natural sources and can be classified as Kampo products or non-Kampo products. Unlike non-Kampo products which are folk medicines that lack particular school of thought or the foundation of TM principles [50], Kampo products derive from Kampo medicine principles that originated from TCM (with Shang Han Lun being the most reputed classic textbook). According to WHO, Kampo medicine is defined as “the medicine traditionally practiced in Japan, based on ancient Chinese medicine” [55]. The approval system for Kampo products depends on their regulatory status. For ethical Kampo products (or known as Kampo formulation for prescription), the approvals were granted solely based on chemistry, manufacturing, and control data but not clinical trial data in 1986. Due to the changes in the approval system for ethical Kampo products that imposed the same evaluation standards as for new medicines, no new ethical Kampo products have been approved since 1986. For over-the-counter (OTC) Kampo medicines, according to the latest version of “The Guidebook of the Approval Standards for OTC Kampo Products” published in 2017 [56], 294 formulas were listed. Considering that these listed Kampo formulas have been in use over many centuries, no preclinical and clinical data is necessary for product application.

#### 3.1.5. Korea

Although the medical system in Korea is divided into a modern medical system and a Korean traditional medical system, medicines are controlled universally by the Ministry of Food and Drug Safety according to the Pharmaceutical Affairs Act. According to “the Regulation on Approval and Notification of Herbal (crude) Medicinal Preparations, Ect.” [57], to manufacture herbal medicinal products, one must obtain the permission of the drug authority by submitting data on the standards and test methods, safety, and efficacy. For preparations with the same ingredients, dosages, and efficacy that are included in the ten herbal medicine books recognized by the Ministry of Health and Welfare Notification, clinical data on the safety and efficacy of the preparation are exempted [54], as they are regarded as having established in safety and efficacy with the support of traditional literature. For the purpose of this study, we mainly focus on the herbal drug with its prescription adjustment enlisted in the herbal medicine book (but adjustment based on the literature other than the herbal medicine book).

### 3.2. The Listing of Classic Formulas

A catalogue system is in place to verify, review, and revise the listing of TM/CM products to be considered as those with a long history of use. The catalogue of CCMF in China is managed by a project working group composed of TCM professional experts and organized by the State Administration of TCM of China. The working group selected 531 ancient *classic formula*s from more than 100,000 prescriptions of 103 representative medical books before the Qing Dynasty [58]. So far, the first batch of 100 CCMF has been issued under the Selection Scope and Principles [59]. In Taiwan, in order to promote the development and unification of TCM preparations, the Ministry of Health and Welfare compiled a list of 200 SFCM based on the types and frequencies of commonly used TCM preparations and announced them in two batches. With standardized preparations, TCM practitioners will be able to control the dose and efficacy and establish standardized management norms of TCM preparations. In Japan, a list of 210 Kampo formulas was selected from a collection of 700 formulas originally developed by experts from reference texts in the 1970s. The catalogue is mainly to differentiate Kampo formulas that fit the reimbursement scope of Japanese medical insurance system and has been subject to multiple revisions in the past decades. Recently, 84 formulas have been added to the Kampo formulas catalogue as mentioned in “The Guidebook of the Approval Standards for OTC Kampo Products” [56].

Comparison across these catalogues of *classic formula* shows a high level of similarity at least by the name of the formula: 28 *classic formulas* commonly found on China and Japan catalogues, 37 *classic formul*as commonly found on China and Taiwan catalogues, and 89 *classic formulas* commonly found on Japan and Taiwan catalogues. Overall, China, Japan, and Taiwan catalogues have 17 common *classic formulas* (Huanglian Decoction, Ganluyin, Wuzhuyu Decoction, Guizhishaoyaozhimu Decoction, Wenjing Decoction, Wendan Decoction, Dangguiyinzi, Shaoyaogancao Decoction, Xiaochengqi Decoction, Zhenwu Decoction, Qinxinlianziyin, Qinfei Decoction, Dajianzhong Decoction, Zhuling Decoction, Taohechengqi Decoction, Dangguisini Decoction, and Mahuang Decoction). The representative bibliographies of the selected *classic formulas* listed in the catalogues are the records of Shang Han Lun, Jin Kui Yao Lue, He Ji Ju Fang, and Wang Bing Hui Chun and other ancient medical books.

Another important indicator of original provenance is the origin of the *classic formula* which largely refers to a collection of ancient medical textbooks that are considered important indicators of a long-term application process throughout the history of mankind. Korea has listed 10 herbal medicine books as the bibliography of *classic formulas*. Among them, Dong-Eu-Bo-Gam (by Hur Joon, Anno Domini 1713) is the greatest masterpiece and is considered as a bible of Korean traditional medicines up to the present in Korea [60]. Hong Kong states that *classic formulas* are limited to those that have been recorded in the Chinese medicine bibliography in or before the Qing Dynasty, the Chinese Pharmacopeia, or the National Drug Standards of PRC. The bibliography and content of the selected *classic formulas* in the investigated countries and regions are summarized in Table 3.

### 3.3. Registration Requirements and Restrictions

#### 3.3.1. Registration Dossier Requirements

In general, each of the investigated countries and regions offers the simplified registration pathways for TM/CM products featured with a long history of use, which is different from the general full registration pathway for new drug that requires proven efficacy data derived from clinical trials. The essence of the simplified registration is the consideration of the totality of evidence attributed to both clinical data from clinical settings and controlled trials. Although the specific requirements for evidence to demonstrate quality, safety, and efficacy vary across the regulatory systems (as shown in Table 4), there is a common emphasis on quality control. Regarding product safety documents, they can be exempted from submission in Japan and Taiwan, while others need some toxicity test reports.

#### 3.3.2. Registration Restrictions

Although clinical trial data may be exempted when applying for registration of TM/CM products, the countries and regions under investigation impose additional restrictions across the following 7 aspects to supplement the consideration of the totality of evidence and to minimize safety risks.

*(1) Formula Composition*. In China, the inclusion of any ingredients with severe toxicity or restricted use in the CCMF is forbidden. Specific attention is also paid to the herb-herb interactions that might lead to serious unwanted effects or a reduction in the therapeutic effects of the herbal ingredients in cases such as “eighteen antidrugs” and “nineteen fears.”

*(2) Manufacturing Process*. It specified that water is the only solvent that can be used for the extraction of ingredients (crude drugs in Japan or prepared slices of crude drug in China) in the manufacturing process [61]. If other solvents are used in the manufacturing process, pharmacological and clinical trial data will be needed to verify the safety and efficacy.

*(3) Dosage Form*. The choice of dosage forms is required to be based on the traditional preparation recorded from medicine books. In China, except for the granules made from decoctions, other ordinary dosage forms may include powders and ointments. Concentrated preparations such as pills, powders, and ointments are allowed in Taiwan and Japan.

*(4) Administration Route*. The administration routes must be consistent with those recommended in the ancient medical books with oral administration being the main administration route.

*(5) Dosage*. In order to avoid any safety risks caused by excessive intake of the herbal ingredients, the dosage is fixed in Taiwan and Japan. In China and Korea, the recommended dosage must follow what was recorded in the medical textbooks and conversion to appropriate dosage with references and guidelines whenever applicable.

*(6) Medication Safety Information*. Regarding the medication safety information of the product label and package insert, modern medical terms to describe the indication are allowed for the TM/CM products in Japan and Korea, which is not the case in China and Taiwan. For instance, the drug safety information of Kampo medicines is composed of five specific items: warning, taboo, cautions, interaction, and adverse reactions [62], while China requires extra two items, principle basis of functional indication and TCM clinical practice [63].

*(7) Restrictions on the Users*. For the CCMF in China, it is mandated that the user groups should not include those who suffer from emergency, critical illness, or infectious disease, as well as pregnant women, infants, and so forth.

### 3.4. Quality Control

Quality control has a direct impact on the safety and efficacy of products. Despite the registration documents submitted are different, the investigated countries and regions focus on the quality control of products. There are three similarities in quality control of products as follows.

#### 3.4.1. Good Quality Management Practices

All should ensure that the manufacturing procedure of the sales of products complies with Good Manufacturing Practices (GMP). Compliance with Good Agricultural Practices (GAP) is also recommended to help reduce the risks of germplasm confusion and overuse of pesticides and fertilizers in the growing of crude drugs. In China, the application of GAP is encouraged to ensure quality traceability system of medicinal materials which may involve artificial cultivation and breeding. Although Japan has no mandatory requirements from laws and regulations, relevant pharmaceutical associations enacted a self-imposed guideline “Guideline of Cultivation, Collection and Processing of Medicinal Plants” [64] and standard “standards related to production management and quality control of crude drugs and crude drug preparations” [65] to ensure the quality of planting and manufacturing of Kampo medicines.

#### 3.4.2. Hazardous Contaminants Tests

It is a general requirement to test for hazardous contaminants to ensure product safety, including pesticide residues, toxic elements and heavy metals, microorganisms, aflatoxins, and sulfur dioxide residue.

#### 3.4.3. The Establishment of Quality Standards

Among the investigated countries and regions, China, Hong Kong, and Korea specify the standards of the crude drugs which must be included in the application. In China, Taiwan, and Japan, a *standard decoction* or *substance benchmark* is also proposed to serve as the standard reference to measure the consistency between the preparation made under the same formula and the clinically used decoction.

The preparation method of *standard decoction* is prepared by adding 20 times the amount of water to the daily prescription dose of crude drugs, boiling for more than 30 minutes, until the decoction is half the amount of the originally added water [66]. According to the Matters Needing Attention When Approving Applications for Pharmaceuticals (No. 0331009) [67], it is an important task of product quality control to compare the Kampo medicines with the standard decoction. Calculated based on the daily prescription dose of crude drugs, no less than two index components selected from the standard decoction are required for comparison with the corresponding index components of the extract and the final product. Meanwhile, the study data should be provided on at least three batches of the drug products. Each batch must be subjected to testing at least 3 times. Taiwan also referred to the quality control method of “comparative tests with standard decoctions” of Kampo medicines, and a total of 19 standard formulas of Chinese medicines were required to submit quantitative analyses of 2 index components [68].

For the registration of CCMF in China, it is required to submit the research data about the quality of the finished product and the *substance benchmark. Substance benchmark* refers to the standard of medicinal substances in TCM prepared consistent with the preparation methods of *classic formulas* recorded in ancient medical books (except for the molding process) [69]. In detail, the study of *substance benchmark* is to identify and select at least 15 batches of different quality crude drugs from at least 3 producing areas and to prepare corresponding slices of crude drugs according to the processing specifications of ancient medical books and then to make more than 10 batches of *substance benchmark* by following the ancient technical decocting. For the research and development of CCMF products, it is necessary to study the systematic data of quality control from the planting source to the whole manufacturing process of the final product including crude drugs, prepared slices of crude drug, corresponding object of *substance benchmark*, preparation intermediate and final product, and use extract content, assaying of active/index components, fingerprints or characteristic maps as quality indicators. The crude drugs, prepared slices of crude drug, *substance benchmark*, and final product should establish the quality standards, and the detailed items are shown in Table 5.

### 3.5. Postmarketing Monitoring

Each of the investigated countries or regions focuses on the postmarketing monitoring of adverse drug reactions (ADRs) for the regulation of TM/CM products as summarized in Table 6. The spontaneous ADRs reporting system which is a widely used method in postmarket surveillance is in place to collect activities data related to safety. China, Japan, and Korea are members of the WHO Programme for international drug monitoring and their ADRs reporting systems are connected with the WHO Pharmacovigilance Programme [70]. Only Taiwan has an individually operated monitoring system for TM/CM products.

## 4. Discussion

It has been shown in this study that, for TM/CM products featured with a long history of use, the totality of evidence acquired from both practical settings and clinical studies may offer a meaningful approach that leverages regulatory burden and product accessibility, thereby ensuring public health, promoting industry growth, and preserving the culture of TM/CM. While previous attention has been mainly focused on specific exemptions of scientific-based clinical studies, it is the integrated regulatory approach that leads to the leniency for regulators within the prevailing concept of evidence-based medicine. The importance of regulatory standards in quality control and traceability during the premarketing phase and the need for innovative approaches to postmarket surveillance have been universally emphasized across the regulatory systems investigated in this study. There are also additional restrictions in terms of the scope, formula composition, manufacturing method, dosage, dosage form, administration route, medication safety information, and end-users to help safeguard the safety. Critical aspects of the collective approach that regulatory authorities may consider to adopt when evaluating TM/CM products with long-standing use are discussed in the following.

First and foremost, it is important to carefully determine the definition of “a long history of use” according to the historical perspective of traditional indigenous medical practices in the local context when applying to TM/CM products [71]. In this study, TM/CM modalities either indigenous to the local culture (such as TCM in China) or recognized elsewhere may be deemed relevant to the decision-making by the drug regulatory authorities. This is important especially to the usage practice and product availability against the backdrop of internationalization, both people and healthcare choices [72]. Depending on the scope of TM/CM products to be considered, the “history of use” to form the knowledge base may be determined by (1) the documentary record in the literature such as ancient TM literature since a certain time point, the national pharmacopeia, or national monographs, and (2) the history availability of such products in some predefined markets, or both [73]. This formed the catalogue system which should be dynamic by nature due to emerging evidence about safety and efficacy and usage patterns.

A mechanism to monitor, review, and revise the listing of TM/CM products eligible for evaluation based on the totality of evidence should be in place and the decisions made should be informed and communicated with a joint effort involving both regulators and TM/CM expertise (Figure 1). Their responsibilities lie heavily on overseeing the quality of evidence generated during the product development process and the outcomes of clinical use of these products. However, the objectives of protecting and promoting public health and facilitating timely access to quality commercial products and industry growth may easily cause conflicting tensions when deciding on regulatory requirements and evaluation standards. A thorough review of the five regulatory approaches in this study has helped enumerate areas critical for deciding on the stringency which optimize the regulatory outcome about TM/CM products. First, a risk management strategy should start with taking into account the safety profile of individual herbs. Herbs with high risks of severe toxicity, interactions, or other adverse events should be excluded from the permissible list of ingredients for products eligible for simplified registration scheme. The permissible ingredients may be further categorized according to the safety profiles which can then be used to determine the regulatory category of the products (prescription medicine or nonprescription medicines). For instance, the “List of Traditional Chinese Medicine Ingredients for Consumption in Macao” [74], in which herbal ingredients are classified as Group I (toxic medicinal herbal materials), Group II (common medicinal herbal materials), or Group III (medicinal and dietary herbal materials), may serve as a parameter to decide on the regulatory categories (e.g., prescription-only products and OTC products) and the restrictions of health claims to mitigate the risk after the products enter the market.

Another area worth an in-depth deliberation is quality control, stability, and traceability, considering the “complexity” and “variability” of the development process of TM/CM products that spans across planting and production to final clinical application [75]. GAP aims to control various factors affecting the production quality of herbal materials, to standardize various crude drug production processes in order to ensure that the herbal materials are authentic, safe, effective, and consistent in quality [76]. GAP is also an essential means to achieve standardization of the product quality by systematically regulating the production process and controlling the quality of individual herbs. In China and Japan, a comprehensive approach of developing quality standards in the pharmacopoeia and the adoption of GMP and GAP have been shown to be effective in ensuring the quality and safety of TM/CM products [77–79]. Liu et al. [80] proposed that quality markers can explain the authenticity of crude drugs (species, origin, harvesting time, storage and transportation process, and processing methods). Meanwhile, it can grasp the transfer of efficacy substances from *substance benchmark* to final products. However, it remains a great effort to determine the quality markers for herbal medicines and develop quality standards of *substance benchmark* and CCMF product. Research institutes can play an important role in closing the technical gaps so as to support the modernization, standardization, and internationalization of TM/CM. Engaging high performing research institute can also transform the advantages of science and technology into the advantages of supporting effective regulation of TM/CM product and industrial development.

Furthermore, effective pharmacovigilance is a key approach for the monitoring and evaluation of drugs after marketing. Even if the *classic formulas* listed in the catalogue management have been widely in use, their batch-to-batch safety and efficacy warrant close monitoring. The countries or regions under investigation mainly adopt ADRs monitoring. However, the current ADRs monitoring and reporting system is taking a rather passive stance which can hardly provide full support in the detection and evaluation of any adverse reactions should they happen. Proactive pharmacovigilance is a key monitoring approach across the product lifecycle [81]. According to the pharmacovigilance system applied to pharmaceutical products, the utilization of healthcare databases has gradually been incorporated into the ADRs data sources to foster the postmarketing monitoring measures [82–85]. In fact, drug regulatory authorities have been exploring the application of big data in pharmacovigilance [86]. Sentinel is a classic example of postmarketing monitoring system developed by the U.S. Food and Drug Administration in 2008 which collects and pools together data about drug usage by more than 300 million people for high-level analytics [87]. With the advent of the big data era, the innovative strategies of combining real-world study with clinical trials may present as new paths for clinical research and development, as well as clinical effectiveness and safety evaluation, thus supporting drug regulatory decision-making about new product applications as well as indication expansion [88]. In China, the importance of real-world evidence was to fill the research gaps due to the limitations of traditional TCM clinical trials and to address the need for additional evidence to inform policy decisions [89]. Information technology infrastructure and evaluation tools and standards that enable the development of real-world evidence from real-world data to supplement current evidence with human experiences and well-designed observational studies should also be considered as a priority.

Last but not least, the discipline of regulatory science, charged with the objectives to enhance the scientific rationale supporting their benefit/risk analysis and regulatory decisions based on best available science [90], should also be developed and applied to the regulation of TM/CM products [91]. Regulatory science for TM/CM encompasses revolution of operational procedures, advancement in science and technology, and cross-boundary collaborations and facilitates communications and collaboration between drug regulatory authorities and other stakeholders to promote scientific regulation of TM/CM products. China has initiated the “Action Plan on Regulatory Science in China” in 2019 [92] with one of the 9 key areas specifically dedicated to the evaluation of the safety of TM products. Japan has also launched a regulatory science initiative aiming to standardize evaluation approaches across different regulatory agencies [93]. One of the most important outputs of adopting regulatory science by the drug regulatory authorities was extensive active cooperation networks with different stakeholders related to the development of TM/CM products. Cooperation with universities and research institutes is the pathway to resolve any technical challenges in evaluation and regulation. Based on the experiences in China and Japan [91, 93], formulating and providing regulatory training programs is also the core to enhancing the regulatory capacity and facilitating stakeholder communication.

There were some limitations to this study. Taking into account the complexity of drug regulation and evaluation, the brief overview and comparison of the 5 regulatory approaches in this paper are less than sufficient to fully identify and explain the regulatory paradigm applicable to TM/CM products featured with a long history of use. However, the paper findings may be used to initiate the discussion about the critical path when designing and deciding on the regulatory standards and approaches in countries and regions with such needs. Moreover, the investigation of only 5 regulatory systems might have unbalanced focus on Asian oriented TM/CM modalities limiting the findings about the regulation of the overall TM/CM perspectives. We have tried to supplement the findings with the scoping review of literature in English and Chinese to help illustrate the regulation concerns towards related TM/CM products across the world. Despite the limitations, the study provided a detailed spectrum of regulatory enforcement for the registration of TM/CM products with a long history of use and explained the implications of a comprehensive approach which supplement the expedited registration pathway of TM/CM products with a long history of use.

## 5. Conclusion

Expectations about the quality, safety, and efficacy are rising along with the productivity endeavor in the TM/CM industry presenting critical challenges to drug regulatory authorities. The regulatory systems investigated in this study allow less stringent registration requirements for TM/CM products featured with a long history of use, assuming safety and efficacy to be plausible based on historic use. Considering that the quality of TM/CM products will have a direct impact on controlling and monitoring the safety and efficacy of these products, regulatory standards should emphasize the technical requirements for quality control and postmarket surveillance.

## Figures and Tables

**Figure 1:** The close-loop catalogue system for TM/CM products with a long history of use.

**Table 1:** The official websites and major responsibilities of the drug regulatory authorities.

Country/region	Regulatory authority	Major responsibilities
China	National Medical Products Administration (NMPA) (https://www.nmpa.gov.cn)	Supervise the safety of drugs (including traditional Chinese medicines (TCMs)), regulate the registration of drugs, medical devices, and cosmetics, and undertake standards management
	State Administration of Traditional Chinese Medicine (http://www.satcm.gov.cn)	Bear the overall responsibility of the regulation and development of TCMs
Hong Kong	Chinese Medicine Regulatory Office, Department of Health (https://www.cmro.gov.hk)	Provide administrative support and implement regulatory measures
	The Chinese Medicine Council of Hong Kong (https://www.cmchk.org.hk)	Formulate and implement regulatory measures of Chinese medicine
Taiwan	Department of Chinese Medicine and Pharmacy, Ministry of Health and Welfare (https://dep.mohw.gov.tw)	Plan and promote the administration of TCM and its related human resource, healthcare facilities, and quality improvement
Japan	Ministry of Health, Labour and Welfare (https://www.mhlw.go.jp/english/)	Bear the overall responsibility of the improvement and promotion of social security and public health
	Pharmaceuticals and Medical Devices Agency (https://www.pmda.go.jp/english/index.html)	Conduct scientific reviews of marketing authorization application of pharmaceuticals and monitor postmarketing safety
Korea	Ministry of Health and Welfare (http://www.mohw.go.kr/eng/index.jsp)	Coordinate and oversee health and welfare related affairs and policies
	Ministry of Food and Drug Safety (https://www.mfds.go.kr/eng/index.do)	Regulate food, pharmaceuticals, medical devices, and cosmetics

**Table 2:** Comparison of the terminology and description of TM/CM products featured with a long history of use.

	China	Taiwan	Hong Kong	Japan	Korea
*The general concept of TM/CM products*					
Terminology^a^	Traditional Chinese medicines (TCMs)			Kampo medicines	Traditional Korean medicine
Description^a^	The traditional medicine that originated in China and is characterized by holism and treatment based on pattern identification/syndrome differentiation			System of herbal medicine practiced in Japan by both herbalists and practitioners of modern medicine. They are extracts or dry powders made from a mixture of naturally derived herbal medicines. They originated from ancient Chinese medicine and have evolved to the Japanese original style over a long period of time	Medical practice or discipline that is based on the knowledge, cultures, and beliefs of the people of Korea

*The specific concept of TM/CM products with a long history of use*					
Terminology	Classic Chinese medicine formulation	Standard formula of Chinese medicine	Established medicine	Kampo medicine	Herbal drug
	古代經典名方中藥複方製劑	基準方劑	固有藥	漢方製劑	
Description	It refers to the prescription recorded in the ancient Chinese medical book, which is still widely used, with definite curative effect and obvious characteristics and advantages [46]	It refers to a formulation selected and published by drug regulatory authority that has unified specification and determination in the dosage form and formula contents [47]	It refers to (1) an ancient prescription documented in Chinese medicine bibliography in, or before, the Qing dynasty; (2) a modified ancient prescription based on an ancient prescription with reasonable and rational modifications; (3) a pharmacopoeia prescription documented in the Pharmacopoeia of PRC; or (4) any other prescriptions originating from the National Drug Standards of the PRC and accepted by the Chinese Medicines Board [48]	It refers to traditional Japanese herbal medicine used in Japan for more than 1500 years [49]. It includes ethical Kampo formulations and OTC Kampo formulations [50]. Ethical Kampo formulation is synonymous with Kampo formulation for prescription.	It refers to plant-derived materials and preparations with therapeutic or other human health benefits, which contain either raw or processed ingredients from one or more plants, inorganic materials, or animal origin [51]
Regulatory agency	National Medical Products Administration of China	The Department of Chinese Medicine and Pharmacy, the Ministry of Health and Welfare	(1) Registration authority: Chinese Medicine Council of Hong Kong, Chinese Medicine Division of the Department of Health (2) Postmarketing: Drug office of the Department of Health	The Ministry of Health, Labour and Welfare; the Pharmaceuticals and Medical Devices Agency	Ministry of Food and Drug Safety of Korea (1) Market authorization: Herbal Medicine Product Division, Biopharmaceuticals and Herbal Medicine Bureau (2) Registration authority: Herbal Medicines Products Division, Biopharmaceuticals and Herbal Medicines Evaluation Department
Legislation	Law of the People's Republic of China on Traditional Chinese Medicine, 2016; Pharmaceutical Administration Law, 2019; Provisions for Drug Registration, 2020; Administrative Regulations on Simplified Registration Evaluation and Approval of Classic Chinese medicine Formulation, 2018	Chinese Medicine and Pharmacy Development Act, 2019; Pharmaceutical Affairs Act, 2018; Regulations for Registration of Medicinal Products, 2020; the Regulation on the Preparations of Inherited Formulation and Over-the-Counter Drugs, 2018	The Chinese Medicine Ordinance (Cap. 549 of the Laws of Hong Kong), 1999	Pharmaceutical Administration and Regulations in Japan, 2020; the Guidebook of the Approval Standards for OTC Kampo Products, 2017	Pharmaceutical Affairs Act, 2016; Regulation on Safety of Pharmaceuticals, 2018; Regulation on Approval and Notification of Herbal (Crude) Medicinal Preparations, 2015

^a^The terminology TM/CM was retrieved from the medical subject headings (MeSH) of PubMed.

**Table 3:** Comparison of the listing of *classic formulas*.

	Classic Chinese medicine formulation (China)	Standard formulation of Chinese medicine (Taiwan)	Established medicines (Hong Kong)	Kampo medicines (Japan)	Herbal drugs (Korea)
Legal warrant of the selected *classic formulas*	First Batch of Classic Chinese Medicine Formulas Catalogue	(1) Announcement No. 84056272 of drug Manufacturing of Department of Health; (2) Announcement No. 89037929 and No. 0900002545 of Chinese Medicine Committee of Department of Health	Registration of Proprietary Chinese Medicines	The Guidebook of the Approval Standards for OTC Kampo Products	Regulation on Approval and Notification of Herbal (Crude) Medicinal Preparations, etc.
The amount of the selected *classic formulas*	100 (first batch issued)	200	Not specified	294	Not specified
The representative bibliography of the selected *classic formulas*	Originated from 37 ancient medical books, including Shang Han Lun, Jin Kui Yao Lue, Jing Yue Quan Shu, Wen Bing Tiao Bian, Fu Qing Zhu Nv Ke, Yi Zong Jin Jian, Lan Shi Mi Zai, Wang Bing Hui Chun, Tai Ping Hui Min He Ji Ju Fang, et al.	Shang Han Lun, Jin Kui Yao Lue, Tai Ping Hui Min He Ji Ju Fang, Yi Fang Ji Jie, Yi Zong Jin Jian, Wang Bing Hui Chun, Wai Ke Zheng Zong, et al.	Chinese medicine bibliography in or before the Qing Dynasty, PRC Pharmacopoeia, National Drug Standards of PRC	Shang Han Lun, Jin Kui Yao Lue, He Ji Ju Fang, Wang Bing Hui Chun, Ji Sheng Fang, Wai Ke Zheng Zong, Ming Yi Zhi Zhang, Pi Wei Lun, Qian Jin Fang, et al.	Donguibogam, Bangyakhapyeon, Hyangyakjipsungbang, Kyungakjeonseo, Uihakipmun, Jaejungshinpyeong, Kwangjaebigeop, Donguisoosebowon, Bonchogangmok, and “Provision on Types of Herbal Drug Prescription and Preparation Method”
The characteristic of each selected *classic formula* in the catalogue	Original provenance (including description of TCM for functional indication), prescription component, preparation method, usage (definite quantity), and dosage form	Original provenance, prescription component, dosage, dosage form, indication, and precaution	Not specified	Crude-drug component, dosage and administration, and indication	Not specified

**Table 4:** Comparison of the registration dossier requirements.

	The item of major registration documents	Classic Chinese medicine formulation (China)	Standard formulation of Chinese medicine (Taiwan)	Established medicine (Hong Kong)	Kampo medicine (Japan)	Herbal drug (Korea)
(1) General documents	(1.1) Origin or background of discovery, conditions of use in foreign countries	×	×	×	×	◯
	(1.2) The therapeutic group, comparisons with other drugs, and related information	×	×	×	◯	◯

(2) Product quality documents	(2.1) Quality data on crude drugs					
	(2.1.1) The production information of crude drugs	◯	×	×	×	×
	(2.1.2) The resource evaluation of crude drugs	◯	×	×	×	×
	(2.1.3) Quality standards study data of crude drugs	◯	×	×	×	◯
	(2.1.4) Quality standards	◯	×	◯	×	◯
	(2.1.5) Test report	◯	×	◯	×	◯
	(2.2) Quality data on prepared slices of crude drug					
	(2.2.1) Processing information	◯	×	×	×	×
	(2.2.2) Quality standards study data of crude drugs	◯	×	×	×	×
	(2.2.3) Quality standards	◯	×	×	×	×
	(2.2.4) Test report	◯	×	×	×	×
	(2.3) Quality data on corresponding objects of substance benchmark	◯	×	×	×	×
	(2.4) Manufacturing method data of the product					
	(2.4.1) Study data on manufacturing method in each step	◯	×	×	×	◯
	(2.4.2) Manufacturing verification or recorded data	◯	◯	×	×	×
	(2.4.3) Description of manufacturing method	◯	◯	◯	×	◯
	(2.5) Quality data on product					
	(2.5.1) Quality standards study data	◯	△	×	◯	◯
	(2.5.2) Quality standards	◯	◯	◯	◯	◯
	(2.5.3) Test report	◯	◯	◯	◯	◯
	(2.6) Stability test report	◯	◯	◯	△	◯
	(2.7) Data for container and packaging material	◯	×	×	×	◯

(3) Product safety documents	(3.1) Acute, subacute, and chronic toxicity, teratogenicity, and another type of toxicity					
	(3.1.1) Single-dose toxicity test report	◯	×	◯	×	◯
	(3.1.2) Repeated-dose toxicity test report	◯	×	◯	×	△
	(3.1.3) Genotoxicity test report	×	×	×	×	×
	(3.1.4) Local irritation test report	×	×	◯	×	△
	(3.1.5) Carcinogenicity test report	△	×	×	×	×
	(3.1.6) Reproductive toxicity test report	△	×	×	×	×
	(3.1.7) Other toxicity tests	×	×	×	×	×
(4) Product efficacy documents	(4.1) Reference materials on product efficacy	◯	×	◯	×	×
	(4.2) Absorption, distribution, metabolism, and excretion study	×	×	×	×	×
	(4.3) Pharmacodynamic study (primary and secondary)	×	×	×	×	×
	(4.4) Pharmacological study	×	×	×	×	×
	(4.5) Clinical trial report	×	×	×	×	×

○: data submission is required; △: data submission to be required is case-based; ×: data submission is exempted.

**Table 5:** The quality standard items of CCMF product in China.

	Quality standard items
Crude drugs	Base source, medicament portions, origin, harvest time, origin processing, description, identification test, extract content, assaying of active/index components, loss on drying, fingerprint or characteristic spectrum, impurities, pesticide residues, heavy metals and harmful elements, fungal toxins, and other exogenous contamination limits
Prepared slices of crude drug	Source of herbs, base source, description, identification test, extract content, assaying of active/index components, loss on drying, fingerprint or characteristic spectrum, pesticide residues, heavy metals and harmful elements, fungal toxins, and other exogenous contamination limits
Substance benchmark	Description, identification test, extract content, assaying of active/index components, fingerprint or characteristic spectrum, toxic ingredients assaying, loss on drying, and other test items
Final product	Description, identification test, loss on drying, assaying of active/index components, extract content, exogenous contamination limits, fingerprint or characteristic spectrum, and other test items

**Table 6:** Comparison of adverse drug reactions (ADRs) monitoring system for TM/CM products.

	China	Taiwan	Hong Kong	Japan	Korea
Major ADRs monitoring agency	(1) National center: National Center for ADRs Monitoring, China Center for Drug Reevaluation; (2) Regional centers: each province has its regional center	The Department of Chinese Medicine and Pharmacy, the Ministry of Health and Welfare	Drug Office, the Department of Health	The Ministry of Health, Labour and Welfare; the Pharmaceuticals and Medical Devices Agency	(1) National center: Korea Institute of Drug Safety & Risk Management; (2) Regional centers: the Regional Pharmacovigilance Center
Technical system for ADRs reporting	Direct Reporting System of ADRs	Taiwan ADRs Reporting System for TCM	ADRs Online Reporting	ADRs and Infection Reporting Systems	Decentralized Pharmacovigilance System, National Pharmacovigilance Network
ADRs reporter	Pharmaceutical companies, hospitals, pharmacies, drug distributors, and marketing authorization holders	Medical care institutions, pharmacies, and license holders of all approved medical products	Healthcare professionals and pharmaceutical industry	Manufacturers and healthcare professionals	Pharmacies and hospitals, pharmaceutical companies
A member of the WHO Programme	Y	N	N	Y	Y
Included in spontaneous ADRs reporting system	Y	Y	Y	Y	Y
the ADRs monitoring for TM/CM product	Y	Y	Y	Y	Y
Disclosed ADRs reports on TM/CM product	Y	Y	Y	Y	N

Y: yes; N: no.

## Data Availability

The data supporting the findings of the study are available from the corresponding author upon request.

## Abbreviations

TM: Traditional medicine
CM: Complementary medicine
TCM: Traditional Chinese medicine
TCMs: Traditional Chinese medicines
SAR: Special administrative region
CCMF: Classic Chinese medicine formulation
WHO: World Health Organization
MeSH: The medical subject headings
NMPA: National Medical Products Administration
PRC: The People's Republic of China
SFCM: Standard formulation of Chinese medicine
OTC: Over-the-counter
GMP: Good Manufacturing Practices
GAP: Good Agricultural Practices
ADRs: Adverse drug reactions.
